# Directly Reprogrammed Human Neurons to Understand Age-Related Energy Metabolism Impairment and Mitochondrial Dysfunction in Healthy Aging and Neurodegeneration

**DOI:** 10.1155/2021/5586052

**Published:** 2021-12-14

**Authors:** Camila Gudenschwager, Isadora Chavez, Cesar Cardenas, Christian Gonzalez-Billault

**Affiliations:** ^1^Department of Biology, Faculty of Sciences, Universidad de Chile, Chile; ^2^Geroscience Center for Brain Health and Metabolism (GERO), Santiago, Chile; ^3^The Buck Institute for Aging, Novato, USA; ^4^Universidad Mayor, Center for Integrative Biology, Santiago, Chile; ^5^Department of Chemistry and Biochemistry, University of California, Santa Barbara, USA; ^6^Department of Neurosciences, Faculty of Medicine, Universidad de Chile, Chile

## Abstract

Brain aging is characterized by several molecular and cellular changes grouped as the hallmarks or pillars of aging, including organelle dysfunction, metabolic and nutrition-sensor changes, stem cell attrition, and macromolecular damages. Separately and collectively, these features degrade the most critical neuronal function: transmission of information in the brain. It is widely accepted that aging is the leading risk factor contributing to the onset of the most prevalent pathological conditions that affect brain functions, such as Alzheimer's, Parkinson's, and Huntington's disease. One of the limitations in understanding the molecular mechanisms involved in those diseases is the lack of an appropriate cellular model that recapitulates the “aged” context in human neurons. The advent of the cellular reprogramming of somatic cells, i.e., dermal fibroblasts, to obtain directly induced neurons (iNs) and induced pluripotent stem cell- (iPSC-) derived neurons is technical sound advances that could open the avenues to understand better the contribution of aging toward neurodegeneration. In this review, we will summarize the commonalities and singularities of these two approaches for the study of brain aging, with an emphasis on the role of mitochondrial dysfunction and redox biology. We will address the evidence showing that iNs retain age-related features in contrast to iPSC-derived neurons that lose the aging signatures during the reprogramming to pluripotency, rendering iNs a powerful strategy to deepen our knowledge of the processes driving normal cellular function decline and neurodegeneration in a human adult model. We will finally discuss the potential utilization of these novel technologies to understand the differential contribution of genetic and epigenetic factors toward neuronal aging, to identify and develop new drugs and therapeutic strategies.

## 1. Introduction

Geroscience is an emerging, rapidly evolving field. Modern societies currently enjoy high life expectancies associated with improved healthcare systems and better living conditions. As the world's population ages, it becomes clear that a longer life does not necessarily come hand-in-hand with a healthy life. Like other organs, brain performance, including cognition, emotions, and autonomic functions, declines with age [1]. Aging itself is the leading risk factor in the development of neurodegenerative diseases. Among them are Alzheimer's (AD) and Parkinson's (PD) disease and frontotemporal dementia (FTD) [2]. An accurate and thorough understanding of the molecular, cellular, and physiological aspects compromised during aging will allow us to identify and test novel therapeutic strategies to overcome the harmful consequences of human brain aging.

The possibility of studying human adult neurons obtained by cellular reprogramming strategies represents a novel and advantageous approach to unravel pathways and cellular processes underlying neurodegeneration. Conversion of somatic fibroblasts to induced neurons can be achieved with or without an intermediate pluripotent stage, and the obtained neurons are induced pluripotent stem cell- (iPSC-) derived neurons and directly induced neurons (iNs), respectively. iNs retain age-related signatures from the donor fibroblasts, including oxidative metabolism damage and mitochondrial dysfunction [3–6], DNA damage, epigenetic and transcriptional profiles, and nucleo-cytoplasm compartmentalization impairments [3–5]. In contrast, iPSC-derived neurons lose features associated with age, described as “rejuvenation” [7, 8]. Energy metabolism impairment is one of the factors related to the development and progression of NDD, characterized by severe alterations in glucose metabolism that start before symptom presentation. Mitochondrial dysfunction contributes to impaired glucose metabolism and is vital to understanding neuronal aging and neurodegenerative diseases at a cellular level. In this review, we have recapitulated the existing evidence that shows that iNs retain age-associated features of the donor and evidence underpinning the relevance of maintaining certain age-related features to accurately model and neurodegeneration. Finally, we will discuss projections and potential uses of iNs to study brain aging and NDD to evaluate pharmacological and dietary interventions' effects and their potential contribution to drug development and patient-specific therapeutic strategies.

## 2. Brain and Neuronal Aging

Like other organs, brain performance, including cognition, emotions, and autonomic functions, declines with age [1] and elderly individuals become increasingly prone to developing neurodegenerative diseases (Figure 1). The human brain exhibits atrophy and shrinking in gray and white matter during normal aging, related to synapse loss, dendritic regression, and neuronal death, as suggested by histological analyses [9]. Recently, vascular brain capillary damage and blood-brain barrier (BBB) breakdown have been proposed as early biomarkers of human cognitive decline during aging independent of the accumulation of classical pathophysiological proteins amyloid-*β* and tau [10]. Moreover, the human brain experiments a reduction in glucose metabolism that aggravates during the onset and progression of NDDs [11]. NDD-related glucose hypometabolism has been reported to start before symptom presentation and is region-specific; for example, AD is observed in the hippocampus and the entorhinal cortex, while FTD is the frontal and temporal lobe.

Altogether, these molecular changes target two of the main cellular features that nerve cells require to fulfill brain functions: maintenance of neurogenesis and preservation of neuronal network activity [9]. Although the precise contribution of neurogenesis in the human aged brain is still far from being understood, recent advances suggest that newborn neurons are present in neurogenic niches even in octogenarians [12]. In addition, a correlation between a decreased number of neuronal progenitors and Braak stages that mark the progression of AD has been established [12]. To preserve brain activity, neuronal networks encompassing neuronal and glial cells involved in generating synaptic contacts rely on a tight balance between excitatory and inhibitory transmission. It has been proposed that increased excitatory activity is a canonical hallmark of aged brains. Such abnormal behavior is prominently dependent on reduced inhibitory tone as well as increased excitatory transmission [13]. Interestingly, such activity imbalance is also associated with circuit dysfunctions observed in animal models for NDD, such as AD [14, 15].

Brain aging is characterized by neuronal death, synapse loss, and senescence-like phenotypes at a cellular level. The aged brain is characterized by accumulation of organelle dysfunction affecting neuronal nuclei, lysosomes, and mitochondria [9], the accumulation of oxidized macromolecules [16, 17], impaired adaptative responses to stress [18], and deregulated energy metabolism [19] (Figure 1). These changes can, in turn, modify directly or indirectly other relevant cell components such as calcium homeostasis [9] and inflammation [20]. Cellular senescence is one of the hallmarks of aging and is considered a complex phenotype characterized by a state of permanent cell cycle arrest and alterations in morphology and function [21]. Although there is no single marker for senescence, it encompasses common-shared features such as the activation of the senescence-associated lysosomal enzyme *β*-galactosidase (SA-*β*-gal), DNA damage detected by *γ*H2AX foci, expression of cell cycle arrest drivers p16^INK4a^ (Cdkn2a) and p21^CIP^ (Cdkn1a), nuclear deformation due to degradation of nuclear envelope proteins, and the secretion of a distinctive set of molecules, known as the senescence-associated secretory phenotype (SASP) [22, 23]. Using long-term neuronal cultures as a tool has been possible to dive deeper into the specific mechanisms associated with neuronal senescence and the consequences of functional interactions with other cell types in the brain, such as the astrocyte-neuron interaction [24, 25].

In neurons, despite their postmitotic nature, many features of the senescence phenotype, namely, DNA damage, SA-*β*-gal-positive staining, phosphorylated histone *γ*H2AX foci, oxidative stress, and lipofuscin accumulation, have been previously observed in aging mice [26, 27], in culture-aged rat neurons [24, 25, 28] and, some of them, in interneurons derived from fibroblasts of Rett syndrome patients [29] (Figure 1). In a signaling network that has not yet been fully elucidated, reactive oxygen species (ROS) production is also induced by the activation of p21, which together with the metabolic oxidative stress, triggers the DNA damage response that promotes senescence via the induction of p38MAPK and secretion of cytokines such as IL-6 and IL-8 [26]. The study of brain sections is a relevant approach that accounts for aging within the context of a whole organism, allowing the consequences of diet [26] or the extent of vascular damage [30] to be assessed. Nevertheless, such a method is disadvantageous for a more meticulous dissection of cellular and molecular.

In the aged brain, the failure of diverse cellular processes contributes to the physiological decline of neuronal function, exacerbated in neurodegenerative diseases. Deficits in energy metabolism and mitochondrial dysfunction are central features of neurodegeneration (Figure 1); therefore, studying how age alters impairs mitochondrial homeostasis is fundamental to understanding synapse loss and cognitive decline at a cellular level.

## 3. Mitochondrial Function in Brain Aging and Neurodegeneration

### 3.1. Mitochondrial Function and Energy Metabolism in Neurons

In neurons, mitochondria play a fundamental role in synaptic transmission and survival. These organelles are involved in energy metabolism, cell death regulation, calcium homeostasis, and biosynthesis of macromolecules [31–34]. The brain accounts for only 2% of the body mass in humans, mice, and rats, yet receives 20% of cardiac output and glucose, with neurons consuming 75-80% of that energy [35] to maintain the electrochemical gradient across the membrane required for synaptic transmission. Unlike other cell types, neurons rely almost exclusively on the oxidative phosphorylation of glucose mediated by mitochondria to fulfill their energetic requirements. In addition, neuronal mitochondria contribute to Ca^2+^ clearance from the synaptic site, vital for subsequent signal transmission. Mitochondrial function is accompanied by ROS generation, which acts as signaling molecules in normal concentration ranges, but higher levels increase oxidative stress and promote mitochondrial DNA damage [6, 36, 37].

### 3.2. Loss of Mitochondrial Function in Brain Aging and Age-Related Diseases

Because neurons are nondividing cells, they accumulate damage throughout life, leading to mitochondrial function impairments that have deleterious effects in synaptic transmission and network excitability, ultimately promoting synapse loss, cognitive decline, and neurodegeneration [11]. In the aged brain, mitochondrial alterations, such as enlargement and fragmentation [38], impaired electron transport chain (ETC) function [39, 40], increased mitochondria with depolarized membranes [41], and oxidative damage to mitochondrial DNA [42, 43], have been observed (Figure 1). Mitochondrial dysfunction is one of the hallmarks of brain aging and has been extensively associated with glucose hypometabolism during normal aging and NDD. The mechanisms driving altered bioenergetics have not been fully elucidated, and they may be interrelated with mitochondrial dynamics, transport, and mitophagy.

Mitochondrial dynamics are mediated by fission and fusion events that modulate mitochondrial shape and elongation. In neurons, abnormal mitochondrial dynamics are associated with impaired function [44, 45] and contribute to the development of NDDs [46, 47]. Moreover, inhibition of mitochondrial fission rescues energy metabolism and promotes cognitive and motor improvements in AD [48], PD [49], and HD models [50]. Mitochondrial traffic along the microtubules modulates the presynaptic localization of mitochondria, necessary to provide ATP and contribute to Ca^2+^ uptake. In NDD, mitochondria are less motile, and axonal localization is reduced and accumulates in the soma and near the nucleus [51].

Mitophagy is another important phenomenon, a quality control mechanism in charge of retiring damaged organelles and preserving the mitochondrial network [52]. Neuronal mitophagy declines with age, leading to defective mitochondria [53] in axonal swellings and no longer in presynaptic terminals [54]. In hippocampal neurons, mitophagy declines by 70% in old mice compared with young specimens [53]. Similarly, mitophagy is impaired in the hippocampus of AD patients, iPSC-derived human AD neurons, and APP/PS1 mouse models [55]. Mitophagy plays a key role in cellular physiology; however, pathological conditions, including mitochondrial disorders, ischemic stroke, chronic cerebral hypoperfusion, and diabetes, promote excessive mitochondrial disposal that leads to neuronal death, underpinning the duality of mitophagy for neuronal homeostasis and survival [56].

### 3.3. Mitochondrial Dysfunction as a Target for Therapeutic Strategies

Several preclinical studies have targeted mitochondrial function with pharmacological approaches to improve pathological phenotypes of NDDs in mouse models, including mitochondrial division inhibitor [48], complex I inhibitor CP2 [57], and the antioxidant MitoQ [58]. In clinical trials, novel therapeutic strategies aim to improve, preserve, or rescue brain energetics, promote mitochondrial function, target the insulin pathway, or provide alternative fuel sources like ketone bodies [11, 59]. Multiple drugs and metabolites have been reported to restore brain energetics and improve brain function, such as metformin, insulin, glucagon-like peptide 1 (GLP-1) analogs, and ketone bodies. The majority of these drugs target multiple pathways, including mitochondrial function; however, if the modulation of mitochondrial homeostatic processes drives the reported beneficial effects remains to be determined (for more detail, see potential contribution to drug development). In this scenario, a cellular model for adult human neurons is a powerful tool for studying signaling pathways involved in age-related impairments and identifying targets for developing therapeutic strategies.

## 4. The Relevance of a Cellular Model to Study Neuronal Aging and Age-Related Energy Decline

A broad and diverse array of models is being used to uncover the complexity of the aging process, ranging from yeast to animal models (Figure 2). The latter includes invertebrate organisms like *C. elegans* [60] and *Drosophila melanogaster* [61], mammalian organisms including mice [62, 63], nonhuman primates [64], and more recently, and with promising results, companion dogs [65]. These models have been instrumental in identifying evolutionary-conserved aging pathways and modeling brain physiological aging and neurodegeneration [66]. Nevertheless, results from mammalian models are not always reproducible in humans nor translatable to clinical interventions because they fail to recapitulate the pathophysiology of human NDDs. In addition, outcome-based studies performed in both models and human cohorts represent as they overlook the cellular components and molecular mechanisms involved [67, 68]. So far, invertebrate and mammalian models and outcome-based studies are abundant in the geroscience field, whereas cellular models remain elusive and scarce. Even though *in vitro* cultures have often been underestimated for lacking the whole organism perspective, they might constitute the missing key to precisely identifying cellular and molecular components affecting and driving brain aging and NDD.

The discovery that human somatic cells can be reprogrammed to many cell types, including neurons, neuronal progenitors, and glia, started a new era in modern neuroscience. Reprogramming strategies have been developed to obtain neuronal populations to study neurodevelopment and associated diseases and neurodegenerative diseases. It has been recently reported that downregulation or depletion of the RNA-binding protein PTB (PTBP1) allows direct glia-to-neuron conversion of both isolated astrocytes and *in situ* in the mouse. Astrocytes convert progressively to new neurons that can repopulate endogenous neural circuits, alleviating retinal ganglion cell loss symptoms and dopaminergic neuron loss in PD mouse models [69, 70].

Dermal fibroblasts induced to neurons provide a model of human neurons in different stages of human development, including young, adult, and elderly cellular contexts, that otherwise would be impossible to assess.

## 5. Cellular Reprogramming of Fibroblasts to Neurons

Dermal fibroblasts are somatic cells obtained from a skin sample and reprogrammed to neuronal populations following two main strategies: fibroblasts can be directly converted to neurons [3, 71] or converted to induced pluripotent stem cells (iPSC) and subsequently differentiated to neurons [72, 73] (Figure 2). In both cases, the resulting human neuronal populations express canonical neuronal markers such as Tuj1, Map2, and NeuN and display mature neuronal morphologies and electrophysiological properties similar to those in primary neurons [3, 74].

In 2006, Takahashi and Yamanaka reported that somatic cells could be reprogrammed to iPSCs [73]. Soon after, it was reported that iPSC could be differentiated into different cell types, including neurons and neuronal stem cells [72, 75]. In 2010, Vierbuchen et al. reported direct conversion from mouse embryonic fibroblasts to neurons, bypassing the pluripotent intermediary. Before long, human dermal fibroblasts were successfully converted to iNs using different strategies [3, 76, 77]. In 2015, and for the first time, Mertens et al. reported that iNs retain age-associated features that iPSC-derived neurons lose during the reprogramming to iPSC process [3, 7] and are not recovered during the differentiation neurons [78]. The following sections will compare the advantages and disadvantages of direct conversion vs. iPSC protocol and discuss the age maintenance in iNs.

### 5.1. Skin to Model Neuronal Aging

The skin is affected by the combined effect of genetic (or intrinsic) and environmental (or extrinsic) factors. This organ is composed of an outer and inner layer, the epidermis and dermis, respectively. Dermal fibroblasts seldom proliferate, and they rely on damage repair to survive and, therefore, are less likely to eliminate macromolecular damage through cell division [79], in contrast to epidermal fibroblasts, that constantly shed. Thus, dermal fibroblasts constitute a long-lived population undergoing constant macromolecular damage accumulation, similar to neurons.

They can be cultured from skin samples obtained by a punch that cuts a small skin area ~1 cm^2^. Skin samples can be collected and processed to obtain primary fibroblast cultures from individuals or cohorts of interest. In addition, fibroblast cultures are available and can be requested from cell repositories, such as the Coriell Institute or the Tau Consortium [80], where fibroblasts from NDD patients, either sporadic or carrying disease-related mutations.

### 5.2. Directly Induced Neurons

Direct reprogramming, also known as transdifferentiation, converts fibroblasts to neurons directly, without a pluripotent intermediary. Mouse embryonic fibroblasts were directly converted to neuronal populations by expressing the transcription factors *Ascl1*, *Brn2*, and Myt1l [71]. Subsequently, human dermal fibroblasts were successfully converted to neuronal cells by expressing *Ascl1* combined with a small molecule cocktail [81]. Multiple approaches have been developed over the years to obtain specific neuronal cell types and increase conversion efficiency. Among them are neuronal transcription factor (TF) overexpression [71, 82], TF overexpression combined with small molecules [3, 81], microRNA expression [76], and small molecule-based [77, 83] protocols. Depending on the experimental setting, it is possible to obtain mainly glutamatergic, mixed, or cell-specific-type populations as motor neurons [5, 84]. In comparison, directly reprogrammed neurons are more cost-efficient than iPSC-derived neurons because they require less time to be obtained. However, in contrast to clonally expanded iPSCs, iNs are generated from primary fibroblast cultures that can be grown by a limited number of passages, representing a limitation of this strategy [85].

### 5.3. iPSC-Derived Neurons

iPSC-derived neuron protocols involve two main steps: obtention of iPSCs and selection, expansion, and differentiation of an iPSC clone. First, fibroblasts are transduced with plasmids that promote the overexpression of pluripotency-associated transcription factors Oct3/4, Sox2, Klf4, and c-Myc, also known as the Yamanaka factors. The resulting iPSCs exhibit pluripotent features, resembling embryonic stem cells (ESC). iPSCs from colonies that can self-renew and differentiate into cells of the three germ layers. iPSC colonies are selected, clonally expanded, and differentiated using a pharmacological approach that varies depending on the neuronal population of interest [74]. They have been instrumental in studying neuronal development and associated neuronal diseases. Since clonal expansion eliminates the heterogeneity between cells that could interfere in the results, iPSC-derived neurons are especially advantageous for dissecting a particular mutation's contribution to pathology. In addition, genome editing techniques, including CRISPR-Cas9, allow revert mutations and generate homozygous or heterozygous cell populations in an isogenic background. However, this strategy involves more extended culture periods and, overall, is considered an expensive technology. More importantly, there is evidence that the induction of pluripotency in adult fibroblasts promotes changes in epigenetic signatures, erasing age-associated marks and experimenting “rejuvenation” to an embryonic stage [7, 86] independent of the fibroblast donor biological age, making iPSC-derived neurons from old and young donors indistinguishable (Figure 3).

## 6. iNs Retain Age-Associated Signatures from the Fibroblast Donor

It is widely accepted that aging is the leading risk factor contributing to the onset of the most prevalent pathological conditions that affect brain functions, including tauopathies such as AD and FTD, PD, and HD. In this section, we will summarize the evidence supporting that iNs exhibit age-related phenotypes from the donor fibroblasts, including DNA damage, differential epigenetic and transcriptional profiles, altered nuclear architecture, and impaired nucleo-cytoplasmatic transport, with particular emphasis on age-related mitochondrial dysfunction and impaired energy metabolism.

### 6.1. Mitochondrial Metabolism and Oxidative Stress

The most compromised brain regions are the hippocampus and cortical structures in both normal and pathological brain decline. Their neurons are mainly glutamatergic and have the highest activity levels, consuming 80-85% of cellular ATP [87]; thus, they are particularly vulnerable to accumulating oxidative damage leading to functional impairments. There are reprogramming strategies that yield mainly glutamatergic iNs [3, 77], and they have been reported to exhibit damage associated with age and therefore offer a “whole-cell” approach to evaluate neuronal mitochondrial homeostasis *ex vivo* [4, 6] (Figures 3 and 4).

In 2018, Kim et al. reported that iNs derived from old individuals display age-related mitochondrial impairments. They performed an extensive analysis of mitochondria from young and old iNs, including changes in gene expression, morphology, localization, and function [6]. In old iNs, 70% of mitochondrial genes are downregulated, from which 90% are related to complexes I-IV from the electron transport chain (ETC). Mitochondria from old iNs exhibit phenotypes that have been linked with impaired mitochondria: increased fragmentation and reduced length. In addition, the proportion of mitochondria located in axons is diminished. Age-related impairment was assessed at a functional level by measuring mitochondrial membrane potential (*ΔΨm*), intimately related to mitochondrial function. Old iNs have lower *ΔΨm* and consequently lower ATP levels and increased oxidized protein damage [6] when compared with young iNs (Figures 3 and 4). Moreover, iNs derived from old donors exhibit higher levels of ROS [4] and higher oxidative stress [5] than iNs derived from young donors.

In contrast, mitochondria from iPSC-derived neurons experiment “rejuvenation” and a concomitant increase in mitochondrial fitness [78, 88, 89]. The reprogramming process resets mitochondrial structure and functionality to an ESC-like state, restores mitochondrial-associated cell death mechanisms, reduces levels of oxidative stress [88], and raises *ΔΨm* and ATP levels [89].

Furthermore, iNs reflect the heterogeneity of the epigenetic marks of the original fibroblast population and mitochondrial heterogeneity since each iN originates from an individual fibroblast. Unlike iPSC-derived neurons, where all neurons come from one iPSC clone selected to be clonally expanded and ultimately differentiated into neurons.

### 6.2. DNA Damage and Structure

High levels of synaptic activity bring with its accumulation of ROS, which compromises genomic and mitochondrial DNA integrity [90]. Analysis of brain sections from rodents and humans has reported reduced expression and enzymatic activity of proteins involved in DNA repair [91]. Directly induced striatal medium spiny neurons (iMSNs) derived from old individuals (almost centenarian) exhibit higher levels of DNA damage compared to iMSNs derived from postnatal donors [4] (Figure 3). Notably, iPSC-derived neurons from both young and old donors exhibit improved DNA-damage response and restored global heterochromatin [78]. Moreover, in iMSNs, the length of telomeres is unaltered, and it corresponds to the telomere length of the starting fibroblasts, which is related to the donor's age [4]. On the contrary, iPSC-derived neurons restore their telomere size during the reprogramming to pluripotency, and it becomes indistinguishable from those of embryonic stem cells [7, 92].

In another study, old donors' directly induced motor neurons (iMNs) exhibit higher cells *γ*H2AX-positive foci, a canonical marker of senescence, compared to young iMNs. Similarly, old iMN production reduced levels of heterochromatin and loss of nuclear organization, assessed by the levels of LAP2*α*, H3K9me3, and HP1*γ* proteins. Consistent with the reports above, only directly induced MNs exhibit age-related features, while iPSC-derived neurons from the same starting fibroblasts recover nuclear organization and show lower levels of DNA damage [5].

### 6.3. Epigenetic

Changes in transcriptional networks and chromatin state are observed during aging and profoundly affect cellular function and stress resistance, thereby contributing to the progression of aging [93]. It has been reported that the genome becomes globally hypomethylated, except for certain hypermethylated regions [94, 95]. In particular, DNA methylation analysis of 353-specific CpG loci, commonly referred to as the epigenetic clock [94], allows to estimate DNA methylation (DNAm) or epigenetic age and is currently considered the most reliable biomarker correlating biological and chronological aging [96, 97].

In Huh et al., they assessed the epigenetic clock of fibroblasts obtained from individuals ranging from 3 days to 94 years old. They found that the DNAm age of their dermal fibroblasts correlated with their chronological age. Next, fibroblasts were directly induced to iMSNs. Their DNAm age correlated with the corresponding fibroblast DNAm age, strongly suggesting that age-related epigenetic marks are retained and unaltered during the direct conversion [4] (Figure 3). By contrast, it has been documented that iPSC strategies reset the epigenetic clock to an embryonic state since iPSCs have a negative or close to zero DNAm age, which is characteristic of embryonic cells [94]. Notably, even though direct conversion alters the human epigenome and transcriptome to promote changes in cell transcriptional program and cell identity [98], age-related marks appear to be unaltered during the process.

### 6.4. Transcriptional

In the aged brain, genes related to synaptic plasticity and mitochondrial function are affected by DNA damage [91]. On a transcriptomic level, young and old iNs exhibit age-related changes in gene expression. Gene ontology (GO) enrichment analysis showed that differentially expressed genes (DEGs) were related to neuronal function categories, such as regulation of synaptic plasticity, neuron projection development, Ca^2+^ homeostasis, and aging [3] (Figure 3). In a similar study, DEGs were associated with age-related biological processes, including vesicle-mediated transport, nervous system development, regulation of apoptosis, and inflammatory response, among other genes previously identified with brain aging [4]. In contrast, fibroblasts from young and old donors reprogrammed to iPSC-derived neurons display a gene expression profile resembling pluripotent stem cells, with upregulation of Myc-N, Nanog, Oct4, and Otx2, among others, independent of donor fibroblast age [3].

### 6.5. Nuclear Architecture and Nucleo-Cytoplasm Transport

Extensive work has linked defects in nuclear architecture with impaired aging phenotypes. One example is Hutchinson-Gilford progeria syndrome (HGPS), where mutations in the intermediate filament LaminB1, a structural component of the nuclear envelope, promote accelerated aging phenotypes [99]. Moreover, nucleo-cytoplasmatic transport is disrupted in NDDs, including AD, HD, FTD, and normal human aging [100]. Notably, old iNs exhibit nucleo-cytoplasmatic defects, and RanBP17, a nuclear pore-associated transport protein, was found to be significatively downregulated with age in iNs and cortical regions of aged individuals [3].

iNs retain age-associated signatures as they exhibit age-related mitochondrial dysfunction and impairments in oxidative metabolism and genetic, epigenetic, transcriptional, and functional levels. The accumulated effects of aging during life are intimately related to the onset and progression of neurodegenerative diseases; thus, a model that recapitulates the aging signature in a human cellular context will widen our possibilities to understand the mechanisms driving synapse loss, neuronal death, and concomitant cognitive decline.

## 7. Projections and Potential Contributions

### 7.1. Modeling NDD

Recent data highlight the importance of age in modeling brain aging and late-onset neurological disorders, even when studying mutation-driven diseases like HD. It is essential that cellular models truly represent the fitness of mitochondria during aging. Autophagy induction has been widely reported to extend lifespan [62, 101]. However, increased autophagy is detrimental to organismal health when coupled with increased mitochondrial permeability in nematodes and mammals [102]. Higher mitochondrial permeability, one of the features of age-induced mitochondrial dysfunction, was shown to reverse autophagy-dependent extension of lifespan [102].

Primary neurons obtained from mouse and rat embryos have been extensively used to study neuronal development and function. Still, their potential to study age-related phenotypes is limited because they exhibit embryonic phenotypes. An alternative strategy is to culture them for long periods, from 28 up to more than 40 days [28], promoting senescence-like phenotypes (discussed in detail in the brain and neuronal aging). However, the intrinsic differences between mouse and human physiology make it more challenging to translate human brain aging.

As a proxy for neurodegeneration, hippocampal and cortical neurons from wild-type mice are treated with known neurotoxic protein aggregates [48] or obtained directly from mouse models of NDDs carrying pathological mutations [57]. Notably, iPSC-derived neurons from HD patients do not develop mutant huntingtin (mHTT) protein aggregates. They lack a cell death phenotype, despite the expansion of the CAG codon in the gene that encodes for the huntingtin protein (HTT). In contrast, directly induced motor spiny neurons (iMSN) exhibit mHTT aggregates, and mHTT-dependent DNA damage, mitochondrial dysfunction, and spontaneous degeneration in culture over time. It follows that carrying the mutation is insufficient to develop the disease phenotype since the onset and progression require temporal aging itself [84]. Most iPSC-based disease models for NDDs have reported the need to apply additional stress factors to normal culture conditions to elicit disease-specific phenotypes, like ROS or mitochondrial stressors, proteasome inhibitors, and excitotoxic exposure to glutamate, among others [103].

iPSC-derived neurons carrying mutations in the gene coding for tau protein have been developed to study genetic variants of FTD. Similarly, iPSC-derived neurons require long culture periods that range from 30 to 100 days in vitro before they exhibit disease-associated phenotypes [80, 104].

Together, these data underpin the pivotal role of the molecular context that might provide novel insights to complement our current knowledge about the aged human brain and neurodegeneration, even when associated with genetic mutations.

### 7.2. Drug Development

In clinical trials, multiple drugs and metabolites that aim to restore brain energetics in humans have improved brain function and energy metabolism. They include the administration of metformin [105], insulin [106], glucagon-like peptide 1 (GLP-1) analogs [107–109], and ketone bodies [110], among others. In clinical trials, the emerging findings are based on cognitive improvements, while the molecular mechanisms mediating the effects in the aging brain remain poorly understood. The advantages of identifying the molecular mechanisms and targets of such compounds are clear: secondary effects can be avoided by developing new drugs that act specifically on a known site of interest, while drugs already approved by the Food and Drug Administration (FDA) can be repurposed to treat or prevent neuropathological manifestations of NDD [111] (Figure 5).

The majority of these drugs have multiple targets and affect different pathways, including mitochondrial function; however, the specific mechanism that mediates their beneficial effects has not been entirely determined. Metformin has been reported to affect mitochondrial function in multiple manners, including complex I inhibition and diminished ROS production [112, 113], and activation of AMPK [114] that promotes mitochondrial biogenesis [115]. Furthermore, it has been proposed that targeting mitochondrial function might be the primary mechanism of action of metformin [116], driving the beneficial effects on T2D and age-related improvements in life and healthspan, but this remains to be determined. Similarly, GLP1-R agonists have been used to treat diabetes and insulin resistance and based on findings in animal models, their potential to prevent or improve NDDsares being tested [109, 117]. GLP-1 analogs have been reported to improve cognitive outcomes in transgenic models of AD [118, 119] and PD [109]. They enhance mitochondrial function, lower oxidative stress, and reduce proapoptotic mitochondrial signaling. Besides, GLP-1 and their analogs recover mitochondrial damage in pancreatic *β* cells [120] and promote mitochondrial function in brown fat in diet-induced obesity models, at least in part mediated by the AMPK-SIRT-1-PGC1-*α* signaling pathway [121]. In addition, a pilot clinical trial showed that estrogen receptor *β* agonist *(S)-*equol increases cytochrome C oxidase activity in AD [122].

Incorporating iNs into such analyses would be tremendously advantageous. They retain macromolecular damage and epigenetic markers associated with aging yet enjoy the simplicity of a cellular model, compared to brain homogenates, where multiple cell types are present. Thus, we foresee a new scenario where an aged neuronal model might help us discover compounds that directly target the brain and neuronal energetics, similar to the successful use of invertebrate models in stimulating the identification of rapamycin [62].

### 7.3. Mechanisms of Dietary Interventions

Lifestyle interventions, such as caloric restriction, intermittent fasting, ketogenic diet, and fasting-mimicking diet, have proven to extend lifespan and, more importantly, improve healthspan in animal models. Caloric restriction reduces mitochondrial brain aging, including ETC function and overall mitochondrial health, and there is evidence that it can also stimulate mitochondrial biogenesis in neurons [9, 33]. Nevertheless, the molecular mechanisms underlying the beneficial effects of caloric restriction in brain energetics and metabolism in humans have yet to be determined. Similarly, it is unknown whether other dietary interventions might target mitochondrial function directly or indirectly. Therefore, to understand how these treatments affect neuronal function, a model that mimics the metabolic impairment of neuronal cells is required (Figure 5).

### 7.4. Potential Contribution to Precision Medicine

In contrast to controlled laboratory set-ups, humans are exposed to extensive and multiple factors, ranging from diet and lifestyle to geographic and contamination levels. Studies based on the longitudinal observation of twins suggested that only 20-30% of lifespan extension depends on heritable genetic traits [20]. Thereby, epigenetic control of brain functions appears as an essential component to explain overall brain performance and propose strategies that preserve cognitive reserves [123]. As such, genetic and environmental heterogeneity strongly suggest that interventions, dietary or pharmacological, will probably have different results depending on the particular context of each individual. Notably, caloric restriction has no effect in some strains of *D. melanogaster* and mice, suggesting that it depends on genetic and epigenetic contexts [68]. Direct reprogramming allows studying patient-specific iNs, which carry genetic background and the accumulation of environmental stimuli during life. Patient-derived iNs will reflect the metabolic state of the individual; thus, they could be particularly advantageous to evaluate the effects of dietary and pharmacological interventions at a personalized level (Figure 5).

### 7.5. Biomarkers for NDDs

Mitochondrial dysfunction and impaired energy metabolism precede neuronal death and cognitive decline in NDD. There is evidence that cytochrome C activity is decreased in symptomless young adults carrying the APOE4 allele [124] and that expression levels of mitochondrial proteins are diminished in the brains of older people experiencing accelerated cognitive decline [125]. Since iNs reflect the mitochondrial defects associated with age, they might be instrumental in recognizing biomarkers for NDD by studying mitochondrial function in individuals at risk of developing NDDs before and after symptom presentation (Figure 5).

## 8. Conclusions

Normal brain aging and NDDs represent a major socioeconomic, medical, and scientific challenge because they negatively impact the lives of the growing number of individuals who suffer these pathologies and their respective carers. Despite the extensive efforts, there are still gaps in our knowledge of molecular mechanisms driving brain functional decline in humans, and there are no available therapies for NDDs. A cellular model configures human neurons in an aged context might be the missing piece of the puzzle between outcome-based results and histological examination of final stages. The studies conducted in embryonic neurons and iPSC-derived neurons appear to reflect only the initial stages of development. In iNs, the complexity and heterogeneity of human genetic, epigenetic, and environmental factors meet the specificity of each particular individual, strongly suggesting that iNs are indeed a powerful candidate for studying and hopefully counteracting the mechanisms that drive the onset and progression of NDD and those the underlying beneficial effects of pharmacological or dietary interventions, even at a personalized scale.

## Figures and Tables

**Figure 1:** Brain and neuronal aging. The aged brain is characterized by accumulation of organelle dysfunction affecting neuronal nuclei, lysosomes, and mitochondria, accumulation of oxidized macromolecules such as proteins, lipids, and nucleic acids, impaired adaptative responses to stress, and deregulated energy metabolism. These changes end up targeting two of the main cellular features that nerve cells require to fulfill brain functions: maintenance of neurogenesis and preservation of neuronal network activity. At a cellular level, aging leads to synapse loss and neuronal death, which exacerbate NDD. Despite their postmitotic nature, neurons exhibit a senescence-like phenotype. Mitochondrial energy metabolism is key to neuronal function and synaptic transmission and is dysregulated during aging. Morphological and functional alterations have been reported in aging and NDD; however, cellular and molecular mechanisms remain poorly understood.

**Figure 2:** Models to study the brain and neuronal aging. Various models have been vital to identifying evolutionarily conserved aging pathways from yeast to animals and model brain physiological aging and neurodegeneration. Invertebrates, such as C. elegans and Drosophila melanogaster, have played a key role in identifying signaling pathways that modulate aging and brain aging across species. In addition, mammalian models have been extensively used to model physiological aging and neurodegeneration. On the one hand, outcome basis studies represent a black box regarding the underlying cellular mechanisms. On the other hand, results obtained from primary murine cultures or immortalized cell lines have proven not reproducible in humans. In contrast, reprogramming fibroblasts from elderly individuals with or without neurogenerative diseases to iPSC-derived neurons or iNs is an attractive model to study cellular and molecular mechanisms of aging human neurons. iPSC-derived neurons lose epigenetic marks associated with aging, while iNs maintain age-specific features from the donor fibroblasts, including metabolic impairments. Moreover, since they are patient or individual-derived fibroblasts, an individual's genetic and epigenetic aspects are maintained. They can lead towards patient-specific interventions, moving research into the expanding field of personalized and precision medicine.

**Figure 3:** Directly induced neurons (iN) maintain diverse age-related features from the donor fibroblasts. Both neuron types are compared at three different levels: (i) genetic and epigenetic level, which includes telomere restoration or erosion, chromatin organization, DNA integrity, and age-associated epigenetic signatures; (ii) transcriptional and structural level, which includes lack of maintenance of the NDD age-related phenotype and transcriptional features; and (iii) mitochondrial metabolism and oxidative stress, which includes mitochondrial structure and fitness, ROS and ATP levels, and electric transport chain functionality.

**Figure 4:** iNs exhibit age-related mitochondrial impairments. Emerging therapeutic strategies target mitochondrial function and improve neuronal and brain energetics because of their key role in neurodegenerative diseases associated with age. iNs retain age-related mitochondrial impairments, including morphological, functional, and stress-related features, in contrast to other models, such as murine embryonic cultures from disease models or wild-type animals treated with neurotoxic stressors, and also, iPSC-derived neurons, which, in most cases, require additional stressors or more extended culture periods to exhibit age or NDD-associated mitochondrial phenotypes.

**Figure 5:** Projections and potential contributions of iNs. iNs are a human cellular model to study neuronal aging. They retain age-associated signatures that primary mouse neurons lack because of their embryonic origin, and iPSC-derived neurons lose during the reprogramming to the pluripotent intermediary. Thus, they represent a promising strategy to study mechanisms underlying NDD onset and progression. In addition, they can be instrumental in studying the effects of currently known and used drugs, identifying new molecular targets for drug development, and deepening our understanding of the pathways involved in the beneficial effects of dietary interventions. Moreover, they constitute a stage where biomarkers for disease early diagnosis and prevention can be identified. Notably, this strategy is considered a novel and valuable model to perform precision medicine, given that it is a combination of individual-specific genetic background and environmental stimuli experienced during life and aging.
